The article "Observation on the Curative Effect of Massage Manipulation Combined with Core Strength Training in Patients with Chronic Nonspecific Low Back Pain" was retracted in 2023. Reasons: unreliable results or conclusions; lack of ethics approval or compliance; concerns about the data; concerns about the peer review.

# Observation on the Curative Effect of Massage Manipulation Combined with Core Strength Training in Patients with Chronic Nonspecific Low Back Pain

**DOI:** 10.1155/2021/7534577

**Published:** 2021-10-22

**Authors:** Jianfeng Shu, Dong Li, Weijing Tao, Shu Chen

**Affiliations:** ^1^Department of Acupuncture and Massage, Zhejiang Provincial People's Hospital, People's Hospital of Hangzhou Medical College, Hangzhou 310024, Zhejiang, China; ^2^Department of Rehabilitation Medicine, Zhejiang Provincial People's Hospital, People's Hospital of Hangzhou Medical College, Hangzhou 310024, Zhejiang, China

## Abstract

In this prospective study, we used the random number table method to equally divide 141 patients with chronic nonspecific low back pain (CNLBP) who met the inclusion criteria into 3 groups. One group who received massage manipulation therapy was recorded as the manipulation group (*n* = 47), one other group who received core strength training therapy was recorded as the training group (*n* = 47), and the other group who received massage manipulation combined with core strength training was recorded as the combination group (*n* = 47). All the patients were treated for 1w as the course of treatment, with the treatment conducted for 5 d/w for 4 w and 12 w of follow-up. The efficacies of the 3 groups were evaluated after treatment, and the visual analog scale (VAS) scores, Oswestry disability index (ODI) scores, and waist dynamic and static muscle endurance before and after treatment of the 3 groups were compared, and the long-term efficacies of the 3 groups were evaluated combined with the VAS scores at 6 w and 12 w after treatment. Our result was that, after treatment, the total effective rate of the combination group (95.74%) is significantly better than that of the manipulation group (80.85%) and the training group (78.72%) (*P* < 0.05). After treatment, the VAS and ODI scores of the 3 groups significantly decreased, and the waist dynamic endurance and static muscle endurance significantly increased, and the condition of the combination group was significantly improved compared with that of the manipulation group and the training group (*P* < 0.05). At 6w and 12w after treatment, the VAS scores of the manipulation group and training group were increased compared with those at the end of treatment (*P* < 0.05), there was no significant change in the combination group (*P* < 0.05), and the VAS scores of the combination group at 6 w and 12 w after treatment were lower than those of the manipulation group and training group at the same time point (*P* < 0.05). This suggests that the synergistic effect of massage manipulation combined with core strength training in the treatment of CNLBP can effectively alleviate patients' pain and waist dysfunction, enhance dynamic and static muscle endurance, and have significant short-term and long-term effects, which are worthy of promotion.

## 1. Introduction

Chronic nonspecific low back pain (CNLBP) is one of the more common types of low back pain (LBP), accounting for more than 85% of all LBP patients. It refers to the general term for a kind of low back pain in which imaging and laboratory examinations exclude known pathological or disease factors, and the patient's lumbar, lumbosacral, or buttocks have pain and discomfort for more than 3 months, with or without lumbar dysfunction [1, 2]. The disease has a long course and is difficult to be cured; the incidence rate is increasing year by year, and the recurrence rate is also high, which seriously disturbs the daily life and normal work of patients [3, 4]. For the treatment of CNLBP, European and American countries have formulated various clinical diagnosis and treatment guidelines related to low back pain [5–7]. The expert group of the Spine and Spinal Cord Professional Committee of the Chinese Association of Rehabilitation Medicine also formulated the “Expert Consensus on the Diagnosis and Treatment of Acute/Chronic Nonspecific Low Back Pain in China” in 2016 to unify the diagnosis and treatment standards and standardize the treatment plan. In the consensus, drugs, physical therapy, manipulation, and behavioral cognitive therapy are commonly used for the treatment of CNLBP. It can improve the function and mobility of the patient's lumbar spine to a certain extent and reduce pain and disability. However, its curative effect varies greatly, and the recurrence rate of patients is still high. It is urgent to explore a more optimized treatment plan in clinical practice.

Traditional Chinese massage has been used for the treatment of chronic low back pain since ancient times, and in the recent years, it has been recommended by major physician societies at home and abroad as the first choice for treatment. It has the characteristics of effective operation, simple and convenient, economical and safe, but its effect is difficult to maintain, and it is easy to relapse for a long time [8]. Core strength training is an important training method widely used in sports medicine and rehabilitation medicine; it has reliable clinical evidence in reducing pain and improving lumbar function in patients with CNLBP, but the effect is also difficult to sustain when used alone [9, 10]. Based on the above, in recent years, our department has applied massage manipulation and core muscle training to the clinical treatment of CNLBP patients and found that it has a significant effect on improving the short- and long-term efficacy of patients. It is summarized below.

## 2. Materials and Methods

### 2.1. General Data

From April 2018 to September 2020, 141 patients with CNLBP who met the inclusion criteria were divided into 3 groups according to the random number table method. One group who received massage manipulation therapy was recorded as the manipulation group (*n* = 47), one group who received core strength training therapy was recorded as the training group (*n* = 47), and the other group who received massage manipulation combined with core strength training was recorded as the combination group (*n* = 47). The general data in Table 1 of the 3 groups were not statistically different and were comparable (*P* > 0.05).

### 2.2. Diagnostic Criteria

Referring to the “Expert Consensus on Diagnosis and Treatment of Acute/Chronic Nonspecific Low Back Pain in China”, the criteria are: lumbar discomfort symptoms lasting more than 3 months; the pain location being below the costal margin, above the gluteal striae, and after the bilateral midaxillary line; no nerve root involvement symptoms or vertebrae tube stenosis; no specific lesions; with or without waist weakness, waist stiffness, and restricted waist movement; and with or without lower limb pain.

### 2.3. Inclusion Criteria

① Those who met the diagnostic criteria of CNLBP; ② those who had a history of chronic lumbar strain or waist trauma; ③ age 25–50 years old; ④ no obvious abnormalities in imaging examination; ⑤ the course of disease was more than 3 months; ⑥ the visual analogue score (VAS) was greater than 3 points; and ⑦ patients who had an informed and understanding, signed a consent form and met the follow-up conditions.

### 2.4. Exclusion Criteria

① Those who had less than 3 months of uncomfortable symptoms; ② patients with fractures or osteoporosis; ③ patients with lumbar disc herniation, lumbar spinal canal stenosis, space-occupying lesions in the spinal canal, ankylosing spondylitis, and lumbar tuberculosis; ④ patients with neurological, mental illness, malignant tumors, or infectious diseases; ⑤ patients with severe dysfunction of the heart, lungs, liver, and kidney or blood system diseases; ⑥ pregnant and lactating women; and ⑦ patients with poor treatment compliance and unable to cooperate with training.

### 2.5. Treatment Methods

The 3 groups of patients were given health education and posture correction guidance, including paying attention to keeping the waist warm, exercises for strengthening the back muscles; avoiding sitting or standing for a long time; choosing a high chair with backrest when sitting; choosing a hard bed when lying down; heavy objects should be kept as close to the body as possible. At the same time, the therapy group was supplemented with massage therapy, the training group was supplemented with core strength training therapy, and the combined group was supplemented with massage therapy combined with core strength training. 1w was the time period for 1 course of treatment; the treatment was 5 d/w for 4 w, followed by 12 w of follow-up.

Massage manipulation: first, the waist, back, and buttocks are relaxed in a large area by rolling and kneading. This is followed by plucking the first lateral line of the foot sun bladder meridian, pressing on both sides of the spine, and implementing the cross partial pressure method and impact pressure method on the back. Then, the chest expansion traction trigger method, the lumbar spine posterior extension trigger method, the lumbar spine oblique trigger method, the shoulder triggering and waist pushing method, the lumbar spine lifting and shaking method, and other related massage methods are performed. Finally, the rolling method and the false palm slap method were implemented to end the operation. The strength of the whole journey was from light to heavy. For specific methods, please refer to the 2009 edition of “Tuina Manipulation” by Shanghai Science and Technology Press. The time was 20∼30 min.

Core strength training: ① plank support with alternating shoulder touch: the patient took the prone position, first made the plank posture, then touched the opposite shoulder with one hand, and then touched the opposite shoulder with the other hand, alternating bilaterally. 12 times was considered 1 group, likewise 3∼4 groups/day. ② Half body push-ups: the patient took the prone position, supported the upper body with both hands and lifted the upper body off the ground, lifted the head as far as possible and stretched it backwards, kept the pelvis close to the ground, and kept breathing evenly. ③ Hip bridge training: the patient lied on his back with his knees bent, his arms were naturally separated to the sides and laid flat on the ground, the hips were lifted upwards with force, drove the waist and thighs to lift upwards, used feet as one fulcrum, used shoulders and upper back as the other fulcrum, so that the shoulders, abdomen, thighs, and calves were arched like a bridge, and he kept breathing evenly. Each group took 30 s, likewise 3∼4 groups/day.

### 2.6. Observation Indicators

1. Clinical efficacy: Subject to the “Standards for Diagnosis and Efficacy of TCM Diseases.” ①Cured: the symptoms of low back pain disappeared and waist function returned to normal; ②markedly effective: the degree of low back pain is significantly reduced, and the waist function is basically restored; ③effective: the degree of back pain is slightly relieved, and the waist function is slightly restored; ④ineffective: symptoms and waist function have not improved. Total effective rate = (cured + markedly effective + effective) number/total × 100%.
2. Visual analogue scale (VAS) score: VAS was used to evaluate the degree of low back pain before and after the treatment of the 3 groups. The total score was 0∼10 scores, and the score was proportional to the degree of low back pain.
3. Oswestry disability index (ODI) score: The ODI questionnaire was used to evaluate the degree of lumbar spine dysfunction before and after treatment of the 3 groups. This included pain (pain intensity and impact on sleep), individual functions (sitting, standing, walking, and lifting), and personal comprehensive functions (activities of daily living, sexual life, social activities, and outing activities), which is a total of 10 factors. Each factor was 0∼5 scores, and the score was directly proportional to the degree of lumbar spine dysfunction.
4. Back muscle endurance: ① Static muscle endurance: Before and after treatment, the patient laid prone on a supine board, crossed their hands and held head, used the anterior superior iliac spine as the boundary, fixed the lower body, and propped up the upper body parallel to the ground, the stopwatch recorded the maintenance time to evaluate its static muscle endurance. ② Dynamic muscle endurance: The patient first laid prone on an inclined board at a 30° angle, with his legs closed together and immobile, and his hands folded on his chest. With the anterior superior iliac spine as the boundary, the upper body was suspended in the air, the lower back contraction movement was performed to make the body straight, then returned to level. The frequency was 25 times/min, until the patient could not continue to complete the action, and the number of effective completions of the patient was recorded to assess their dynamic muscle endurance.
5. Long-term curative effect: The VAS scores of the 3 groups at 6 w and 12 w after treatment were followed up to evaluate the long-term curative effect.

### 2.7. Statistical Methods

Using SPSS22.0 software, measurement data were expressed as ($\bar{x}$ ± *s*), *F* test was used for comparison between multiple groups, and *t* analysis was performed for pairwise comparison between groups. The count data were expressed in (%), and the *χ*^2^ test was adopted. *P* < 0.05 indicated that the difference was statistically significant.

## 3. Results

### 3.1. Comparison of Curative Effect of 3 Groups

After treatment, the total effective rate of the combination group (95.74%) was significantly better than that of the manipulation group (80.85%) and the training group (78.72%) (*P* < 0.05). There was no significant difference between the manipulation group and the training group (*P* > 0.05), (Table 2).

### 3.2. Comparison of VAS Scores before and after Treatment of 3 Groups

Before treatment, the VAS scores of the manipulation group, training group, and combination group were (5.96 ± 1.12), (6.01 ± 1.04), and (6.04 ± 1.05) scores, respectively. After treatment, the VAS scores of the manipulation group, training group, and combination group were (4.46 ± 1.13), (4.77 ± 1.09), and (3.93 ± 1.04) scores, respectively. After treatment, the VAS scores of the three groups decreased significantly, and the combination group was significantly improved compared with the manipulation group and training group (*P* < 0.05). There was no significant difference between the manipulation group and the training group (*P* > 0.05), (Figure 1).

### 3.3. Comparison of ODI Scores before and after Treatment of 3 Groups

Before treatment, the ODI scores of the manipulation group, training group, and combination group were (32.54 ± 7.36), (32.86 ± 7.19), and (33.07 ± 7.30)%, respectively. After treatment, the ODI scores of the manipulation group, training group, and combination group were (18.98 ± 5.82), (18.53 ± 5.51), and (15.44 ± 4.79)%, respectively. After treatment, the ODI scores of the three groups decreased significantly, and those of the combination group was significantly improved compared with the manipulation group and training group (*P* < 0.05). There was no significant difference between the manipulation group and the training group (*P* > 0.05), (Figure 2).

### 3.4. Comparison of Dynamic and Static Waist Muscle Endurance of 3 Groups

Before treatment, the static waist muscle endurance of the manipulation group, training group, and combination group were (59.63 ± 17.58), (58.21 ± 18.05), and (59.60 ± 17.33) *s*, respectively; the dynamic waist muscle endurance were (19.36 ± 7.89), (20.14 ± 7.61), and (19.74 ± 7.63) times, respectively. After treatment, the static waist muscle endurance of the manipulation group, training group, and combination group were (76.25 ± 14.63), (72.21 ± 15.27), and (85.33 ± 13.65) *s*, respectively; the dynamic waist muscle endurance was (25.38 ± 6.71), (24.64 ± 7.92), and (28.43 ± 7.69) times, respectively. After treatment, the dynamic and static waist muscle endurance in the three groups increased significantly, and that in the combination group improved significantly compared with the manipulation group and the training group (*P* < 0.05). There was no significant difference between the manipulation group and the training group (*P* > 0.05), (Figure 3).

### 3.5. Comparison of the Long-Term Efficacy of 3 Groups

At the end of treatment, the VAS scores of the manipulation group, training group, and combination group were (4.46 ± 1.13), (4.77 ± 1.09), and (3.93 ± 1.04) scores, respectively; 6 w after treatment, the VAS scores of the manipulation group, training group, and combination group were (5.02 ± 0.85), (5.21 ± 0.93), and (4.01 ± 0.70) scores, respectively; 12w after treatment, the VAS of the manipulation group, training group, and combination group were (5.18 ± 0.96), (5.30 ± 0.95), and (3.98 ± 0.97) scores, respectively. At 6 w and 12 w after treatment, the VAS scores of the manipulation group and training group were increased compared with the end of treatment (*P* < 0.05), there was no significant change in the combination group (*P* > 0.05), and the VAS scores of the combination group at 6 w and 12 w after treatment were lower than those of the manipulation group and training group at the same time point (*P* < 0.05), (Figure 4).

## 4. Discussion

CNLBP patients are mostly accompanied by varying degrees of recruitment restriction or morphological changes in the core muscles of the waist and abdomen (multifidus, transversus abdominis, etc.), its main manifestations are poor core muscle strength, decreased waist stability, and changes in the overall stability of the spine, which is also the main pathogenesis of the disease [11–13]. The core strength training implemented in this study is a kind of exercise training performed in the patient's painless state. It includes three main actions: plank support with alternating shoulder touch, half body push-ups, and hip bridge training. In recent years, as one of the important methods for the treatment of low back pain, its role in improving neuromuscular strength has been confirmed [14]. Its mechanism of action may be due to the fact that core muscle strength training can help patients improve the strength and endurance of the core muscles through plank support with alternating shoulder touch and hip bridge training and activate and relax the deep and shallow muscles of the lower back through half body push-ups [15]. Muscle strength training enhances the movement and sensory stimulation of the core muscles, attained the function of improving trunk posture control ability and stabilizing core muscles, which in turn contributes to the restoration of spinal balance and pain relief in patients with CNLBP [16, 17]. In addition, there is also a domestic study on the detection of serum inflammatory factor levels in CNLBP patients who have taken core strength training. It was found that after treatment, the inflammatory level in the patient's body was significantly lower than before treatment. This shows that its mechanism of action may also be related to its promotion of the dissipation of inflammatory substances and the circulation of local lymphatic and blood in the patient's body.

Traditional Chinese massage has a long history of treating chronic low back pain. Recent studies have shown that it also has good application value in improving the symptoms of CNLBP [18]. Modern massage manipulation is a treatment method based on the theory of the viscera and meridians of traditional Chinese medicine, combined with the pathological diagnosis, anatomy, and evidence-based medicine knowledge of Western medicine to diagnose and treat patients. It stimulates and acts on specific acupoints and parts of the human body through different massage manipulation (pushing, holding, pressing, rubbing, rolling, kneading, rubbing, etc.). It can adjust the patient's physiological and pathological status as a whole or in both directions, and ultimately help to dredge the meridians, promote qi and blood circulation, and smooth the joints [19]. Modern medicine also believes that the physical stimulation produced by it can cause a series of physiological and biochemical reactions in the local tissues of the action area and can act on local nerves. Through the relevant adjustment of nerve reflex and body fluid circulation, the patient's physiological response is enhanced, and the secondary overall reaction is caused. Furthermore, it is helpful for the improvement of circulation, separation of adhesions, reduction of inflammation, and correction of facet joint disorders [20, 21]. In the massage manipulation of this study, the patient's back and buttocks are first relaxed in a large area by rolling and kneading, which could help relax muscles and activate blood circulation, relieve muscle spasm and fatigue, enhance muscle activity, and promote blood supply. Then, flicking is applied to the first lateral line of the foot solar bladder meridian, which helped to open the occlusion, move Qi and blood, loosen adhesions, and relieve spasm. The compression method on both sides of the spine, the cross partial pressure method and the impact pressure method on the back help to loosen the muscles and tendons to regulate the tendons, to warm the middle and dispel cold, and to harmonize the qi and blood, etc. The implementation of the chest expansion traction trigger method, lumbar spine posterior extension trigger method, lumbar spine oblique trigger method, shoulder triggering and waist pushing method, lumbar spine lifting and shaking method and other related massage methods, which help to stretch the tendons and veins, smooth the joints, loosen adhesions, help reset, etc.. Finally, the rolling method and the false palm slap method were implemented to end the operation. The force was gradually increased from light to heavy, which helped to establish the patient's tolerance and adaptability. As a result, the patient's muscles that were spasm and tense due to pain could be relieved, local blood circulation could be unblocked, and the nerve could be calmed and inhibited by adjusting the balance of excitement and inhibition of the nervous system, thus contributing to reduce the pain symptoms and improve the lumbar function.

In this study, after treatment, the total effective rate of the combination group (95.74%) is significantly better than that of the manipulation group (80.85%) and the training group (78.72%). After treatment, the VAS and ODI scores of the 3 groups were significantly decreased, and the waist dynamic and static muscle endurance were significantly increased, and the combination group was significantly improved compared with the manipulation group and the training group. At 6 w and 12 w after treatment, the VAS scores of the manipulation group and training group were increased compared with the end of treatment, there was no significant change in the combination group, and the VAS scores of the combination group at 6 w and 12 w after treatment were lower than those of the manipulation group and training group at the same time point. This is partly consistent with the conclusions of related research [22, 23]. The above results collectively suggest that both massage manipulation and core strength training are effective methods for the treatment of CNLBP patients, and both of them can effectively reduce the pain symptoms of patients, improve the lumbar spine movement function, and the endurance of the lumbar muscles, but the short-term and long-term effects of the two are limited when used alone, and the synergistic effect of the combined application of the two will help patients to have a better treatment outcome.

In summary, the synergistic effect of massage manipulation combined with core strength training in the treatment of CNLBP can effectively alleviate patients' pain and waist dysfunction, enhance dynamic and static muscle endurance, and have significant short-term and long-term effects, which are worthy of promotion.

## Figures and Tables

**Figure 1:** Comparison of VAS scores before and after treatment of 3 groups ($\bar{x}$ ± *s*, scores). ^*∗*^Compared with the same group before treatment, *P* < 0.05; ^#^compared with the combination group after treatment, *P* < 0.05.

**Figure 2:** Comparison of ODI scores before and after treatment of 3 groups ($\bar{x}$ ± *s*, %). ^*∗*^Compared with the same group before treatment, *P* < 0.05; ^#^compared with the combination group after treatment, *P* < 0.05.

**Figure 3:** Comparison of dynamic and static waist muscle endurance of 3 groups. (a) Static waist muscle endurance; (b) dynamic waist muscle endurance. ^*∗*^Compared with the same group before treatment, *P* < 0.05; ^#^compared with the combination group after treatment, *P* < 0.05.

**Figure 4:** Comparison of the long-term efficacy of 3 groups ($\bar{x}$ ± *s*, scores). ^*∗*^Compared with the same group at the end of treatment, *P* < 0.05; ^#^compared with the combination group at the same time point, *P* < 0.05.

**Table 1:** Comparison of general information between the control group and the study group.

Category	Manipulation group (*n* = 47)	Training group (*n* = 47)	Combination group (*n* = 47)	*χ* ^2^/*F*	*P*
Male/Female (cases)	28/19	26/21	29/18	0.410	0.815
Age (years old)	38.62 ± 7.67	37.98 ± 7.83	36.23 ± 7.52	1.222	0.298
BMI (kg/m^2^)	21.56 ± 3.05	20.94 ± 2.96	21.61 ± 3.09	0.711	0.493
Disease course (months)	32.28 ± 12.60	31.47 ± 13.22	32.54 ± 12.98	0.087	0.916

Complications (cases)					
High blood pressure	6	9	7	0.754	0.686
High blood fat	2	3	3	0.265	0.876
Diabetes	1	1	2	0.515	0.773
Others	2	2	3	0.301	0.860

**Table 2:** Comparison of curative effect of 3 groups [*n* (%)].

Group	Cured	Markedly effective	Effective	Ineffective	Total effective
Manipulation group (*n* = 47)	5	19	14	9	38 (80.85)^*∗*^
Training group (*n* = 47)	3	21	11	10	37 (78.72)^*∗*^
Combination group (*n* = 47)	12	28	5	2	45 (95.74)
*χ* ^2^					6.379
*P*					0.041

^*∗*^Compared with the combination group, *P* < 0.05.

## Data Availability

The primary data to support the results of this study are available at reasonable request to the corresponding author.
